RETRACTED

# Assessment of Serum Uric Acid Levels Among Gestational Diabetes Patients in Erbil City

**DOI:** 10.7759/cureus.90049

**Published:** 2025-08-14

**Authors:** Lezma G Qadir, Jwan M Zangana

**Affiliations:** 1 Family Medicine, Kurdistan Higher Council of Medical Specialties, Erbil, IRQ; 2 Family Medicine, College of Medicine, Hawler Medical University, Erbil, IRQ

**Keywords:** childbearing age, gestational diabetes mellitus (gdm), high-risk pregnancy, obesity-related illnesses, serum uric acid level

## Abstract

Background and objectives: Gestational diabetes mellitus (GDM) is a common obstetrical disorder with a significant impact on maternal and fetal well-being. This study aimed to assess serum uric acid levels in pregnant women with GDM and determine their diagnostic performance.

Methods: A case-control study was conducted at Erbil Maternity Hospital and primary health care units from May to December 2024, involving 200 pregnant women (100 with GDM and 100 healthy controls). Sociodemographic, obstetric, dietary, and laboratory data were collected. Serum uric acid was measured using the uricase method, and its association with GDM was evaluated using receiver operating characteristic (ROC) curve analysis and multivariable logistic regression.

Results: Serum uric acid demonstrated excellent discriminative ability for GDM (area under the curve (AUC) = 0.940). The optimal cut-off value of 3.15 mg/dL yielded 90% sensitivity and 80% specificity. Women with uric acid ≥ 3.15 mg/dL had 122.8-fold higher odds of GDM (odds ratio (OR) = 122.8, 95% confidence interval (CI): 34.4-437.8, p < 0.001) after adjusting for age, body mass index (BMI), and gestational age; each 1 mg/dL increase was associated with a 30.7-fold increase in odds (OR = 30.7, 95% CI: 10.9-86.3, p < 0.001). Elevated uric acid was present in 90% of women with GDM compared to 11% of controls. This prevalence is higher than that reported in Egypt (54.7%) and India (74.7%). Higher BMI, grand multiparity, positive family history of diabetes, and reduced plant-based food intake were also significantly associated with GDM.

Conclusion: Elevated serum uric acid is strongly associated with GDM, with a cut-off of 3.15 mg/dL providing high diagnostic accuracy. The prevalence observed was higher than in several international studies. Limitations include the facility-based design, lack of adjustment for diet and renal function in the analysis, and potential recall bias.

## Introduction

Gestational diabetes mellitus (GDM) is a pregnancy-related metabolic disorder in which glucose intolerance causes high blood sugar levels in women who have no prior diagnosis of type 1 or type 2 diabetes. In most cases, the condition resolves after delivery [1]. Globally, about 9% of pregnant women are diagnosed with GDM before delivery [2]. In the Middle East and North Africa (MENA) region, the prevalence of GDM is approximately 14% [3], while in Erbil city, Kurdistan Region/Iraq, it has reached 11.9% [4]. This prevalence has increased in recent decades due to sedentary lifestyle, westernization of diet, physical inactivity, and increased maternal body weight. Understanding these prevalence trends is important when considering potential predictive markers for GDM, such as serum uric acid (UA).

RETRACTED

Gestational diabetes commonly develops in the second trimester, although it can occur at any stage of pregnancy [5]. GDM is explained by the pancreas's inability to adjust insulin secretion during pregnancy [6]. Additionally, insulin resistance naturally increases throughout pregnancy and is accompanied by higher insulin secretion; when the maternal pancreas fails to secrete enough insulin, GDM leads to hyperglycemia [7].

Screening and diagnosis of gestational diabetes are important for early treatment due to its adverse effects on both mothers and infants. GDM is associated with early gestational complications such as increased blood pressure, cesarean section, pre-eclampsia, macrosomia, labor difficulties, respiratory distress syndrome, and congenital malformations [8]. In subsequent pregnancies, it may also increase the risk of developing type 2 diabetes [9]. Screening and diagnosis of GDM commonly involve a two-step approach (a 50 g glucose one-hour test followed by a 100 g three-hour oral glucose tolerance test (OGTT)). Nowadays, the 75 g OGTT is used as a one-step technique, offering clinical benefits and helping prevent complications [5].

Serum UA is a product of purine metabolism that increases in various diseases, and its elevated levels have been associated with several adverse gestational outcomes. In normal pregnancy, UA levels typically decrease by 25% to 35% in early gestation and return to pre-pregnancy levels by the end of pregnancy [10]. The possible role of serum UA in the development of GDM has been investigated in various populations, with mixed results. Numerous authors have reported that increased serum UA is linked to metabolic abnormalities, as it inhibits insulin signaling and contributes to the development of insulin resistance [11]. Similarly, other studies have identified high serum UA as a component of metabolic syndrome and insulin resistance [12]. One study found that hyperuricemia may impair endothelial function, resulting in reduced nitric oxide production [13]. Low nitric oxide levels play a major role in the development of hyperglycemia [14]. Moreover, elevated serum UA levels have been associated with insulin resistance in women with gestational hypertension [15]. A previous study reported higher serum UA levels in pregnant women with GDM compared to women without GDM [16]. However, several studies have failed to identify a clear relationship between serum UA and GDM across different trimesters of pregnancy [17]. These discrepancies may be explained by differences in study design, timing of UA measurement, population characteristics, and the diagnostic criteria used for GDM.

RETRACTED

The relationship between serum UA and GDM remains understudied in Iraq, particularly in Erbil, where variations in genetic, dietary, and lifestyle factors may influence this association. Assessing serum UA levels among pregnant women with GDM in Erbil could provide valuable insights into its potential role as an early biomarker, aiding in risk stratification, timely intervention, and improved pregnancy outcomes. The aim of this study was to assess serum UA levels in pregnant women with GDM and identify factors associated with hyperuricemia in this population.

## Materials and methods

A case-control study was implemented in the Diabetic Unit of Erbil Maternity Hospital and the primary health care units of families in Erbil city, Kurdistan Region/Iraq, over a duration of eight months from May 1, 2024, to December 31, 2024. All pregnant women with GDM during the study duration were in the study population. Singleton pregnancies at the second or third trimester of gestation diagnosed with GDM were included. The exclusion criteria were women with a known or past history of hyperuricemia, women on drugs that elevate serum UA levels, women with gestational hypertension in the current pregnancy, women with a history of pre-gestational diabetes, liver and/or renal disease, any other medical disease or condition having an adverse effect on the current pregnancy, and women who did not provide informed consent. Ethical approval of the study was obtained from the Kurdistan Board of Medical Specialties-Research Protocol Ethical Committee, and informed consent was obtained from all participants.

This study included 200 pregnant women divided into two study groups (100 pregnant women with GDM and 100 healthy pregnant women). To determine the appropriate sample size, we assumed a significance level of 5%, a power of 80%, an expected odds ratio (OR) of 2.5, and that approximately 23.7% of non-GDM pregnant women have elevated serum UA levels [18]. Using standard formulas for unmatched case-control studies, the calculated sample size required to detect a statistically significant association was 89 cases and 89 controls. To accommodate potential dropouts or missing data, we rounded the numbers up to 100 in each group for better results. Controls were chosen after confirming that they did not have GDM while attending the primary health care center.

RETRACTED

Women's data were gathered by the researcher directly from the selected women and recorded using a prepared questionnaire designed by the researchers. Content validity was reviewed by two senior faculty members in family medicine and obstetrics. A pilot study was then conducted with 10 pregnant women at a primary health care center to assess clarity, comprehension, and time required for completion. Feedback from the pilot was used to make minor wording adjustments before implementing the questionnaire in the main study. Data from the pilot participants were not included in the final analysis. The questionnaire contained sociodemographic characteristics of study participants (age, residence, blood group, educational level, income categorized as sufficient or insufficient based on the socioeconomic status (SES) index developed by Omer et al. [19], occupation, and house ownership), general characteristics (body mass index (BMI), parity, miscarriage, gestational age (by the last menstrual period (LMP)), family history of diabetes mellitus, weight of previous baby, and food type), and laboratory investigations (random blood sugar level, HbA1c level, serum UA level, and glycosuria). Some patients were diagnosed with GDM upon their first visit to the diabetic unit, and some of them were diagnosed in primary health centers through their antenatal visits. Women meeting the American Diabetes Association (ADA) criteria for overt diabetes in pregnancy (fasting plasma glucose ≥ 126 mg/dL, two-hour plasma glucose ≥ 200 mg/dL, or HbA1c ≥ 6.5% at diagnosis) were excluded [20].

The investigations were implemented in the Laboratory of the Maternity Hospital. A sample of 5 mL of venous blood was drawn from the median cubital vein of all the women. Serum UA was measured by the colorimetric assay, Uric Acid Uricase method (BIOLABO, Italy). GDM was diagnosed based on the one-step approach using a 75 g OGTT, as recommended by the ADA [8]. Data were analyzed using the Statistical Package for the Social Sciences (SPSS) version 26 (IBM Corp., Armonk, NY, US). Categorical variables were compared using the Chi-squared test or Fisher’s exact test, and continuous variables were analyzed with the independent sample t-test. Receiver operating characteristic (ROC) curve analysis was performed to determine the optimal cut-off value of serum UA for predicting GDM, using Youden’s index to identify the point with the highest combined sensitivity and specificity. In addition, multivariable logistic regression analyses were conducted to adjust for potential confounders, including age, BMI, and gestational age. Serum UA was analyzed both as a continuous variable and as a categorical variable based on the ROC-derived cut-off value. ORs with 95% confidence intervals (CIs) were calculated, and a p-value ≤ 0.05 was considered statistically significant.

RETRACTED

## Results

In this study, 200 pregnant women were included. The majority were aged 18-35 years, accounting for 150 women (75%), followed by 49 women (24.5%) aged over 35 years, and only one woman (0.5%) was under 18. Most participants resided in urban areas, comprising 157 women (78.5%), while 43 women (21.5%) lived in rural settings. Regarding education, 87 women (43.5%) were illiterate, and 88 women (44%) had only primary education. Smaller numbers had intermediate education, 13 women (6.5%); secondary education, seven women (3.5%); and college or higher education, five women (2.5%). In terms of income, 169 women (84.5%) reported sufficient income, whereas 31 women (15.5%) reported insufficient or marginally sufficient income. The vast majority were housewives, 175 women (87.5%), followed by 10 non-governmental employees (5%), eight governmental employees (4%), and seven students (3.5%). With respect to housing, 79 women (39.5%) owned their homes, 66 women (33%) lived in partially owned homes, and 55 women (27.5%) resided in rented or other types of housing (Table 1).

**Table 1:** Demographic characteristics of the study population

Variable	n (%), n = 200
Age	
<18 years	1 (0.5%)
18-35 years	150 (75%)
>35 years	49 (24.5%)
Residence	
Rural	43 (21.5%)
Urban	157 (78.5%)
Educational level	
Illiterate	87 (43.5%)
Read, write, & primary	88 (44%)
Intermediate	13 (6.5%)
Secondary	7 (3.5%)
College and above	5 (2.5%)
Income	
Not sufficient, marginally sufficient	31 (15.5%)
Sufficient	169 (84.5%)
Occupation	
Housewife	175 (87.5%)
Student	7 (3.5%)
Governmental employee	8 (4%)
Non-governmental employee	10 (5%)
House ownership	
Rented and others	55 (27.5%)
Partially owned	66 (33%)
Owned	79 (39.5%)

The women in this study were divided into two study groups (100 pregnant women with GDM and 100 healthy pregnant women). Increased age of pregnant women was significantly related to GDM (p = 0.005). There was a highly significant association between illiteracy among pregnant women and GDM (p < 0.001). No significant differences were observed between the study groups with regard to residence, blood groups, income, occupation, and house ownership (p > 0.05) (Table 2).

**Table 2:** Distribution of women's sociodemographic characteristics according to study groups Calculated by the Chi-squared test S: significant; NS: not significant; GDM: gestational diabetes mellitus

Variable	Study groups		Χ^2^	p
	GDM	Control		
	No. (%)	No. (%)		
Age			10.5	0.005^S^
<18 years	0 (0%)	1 (1%)		
18-35 years	66 (66%)	84 (84%)		
>35 years	34 (34%)	15 (15%)		
Residence			3.5	0.058^NS^
Rural	27 (27%)	16 (16%)		
Urban	73 (73%)	84 (84%)		
Blood groups			4.4	0.2^NS^
A	47 (47%)	33 (33%)		
B	18 (18%)	23 (23%)		
O	29 (29%)	34 (34%)		
AB	6 (6%)	10 (10%)		
Educational level			20.4	<0.001^S^
Illiterate	59 (59%)	28 (28%)		
Read, write, & primary	33 (33%)	55 (55%)		
Intermediate	4 (4%)	9 (9%)		
Secondary	3 (3%)	4 (4%)		
College and above	1 (1%)	4 (4%)		
Income			0.8	0.8^NS^
Not sufficient, marginally sufficient	15 (15%)	16 (16%)		
Sufficient	85 (85%)	84 (84%)		
Occupation			1.6	0.6^NS^
Housewife	88 (88%)	87 (87%)		
Student	2 (2%)	5 (5%)		
Governmental employee	4 (4%)	4 (4%)		
Non-governmental employee	6 (6%)	4 (4%)		
House ownership			2.0	0.36^NS^
Rented and others	28 (28%)	27 (27%)		
Partially owned	37 (37%)	29 (29%)		
Owned	35 (35%)	44 (44%)		

Increased BMI of pregnant women was significantly related to GDM (p < 0.001). There was a significant association between grand multiparity of pregnant women and GDM (p = 0.002). A positive family history of GDM was significantly related to GDM (p = 0.002). A significant association was observed between the lack of plant-based food consumption and GDM (p = 0.04). No significant differences were observed between study groups with regard to miscarriage, gestational age, and weight of previous baby (p > 0.05) (Table 3).

RETRACTED

**Table 3:** Distribution of women's general characteristics according to study groups Calculated by the Chi-squared test S: significant; NS: not significant; GDM: gestational diabetes mellitus; DM: diabetes mellitus

Variable	Study groups		Χ^2^	p
	GDM	Control		
	No. (%)	No. (%)		
Body mass index			39.3	<0.001^S^
Underweight	0 (0%)	2 (2.0%)		
Normal	6 (6.0%)	30 (30.0%)		
Overweight	37 (37.0%)	49 (49.0%)		
Obesity grade I	41 (41.0%)	15 (15.0%)		
Obesity grade II	14 (14%)	4 (4%)		
Obesity grade III	2 (2.0%)	0 (0%)		
Parity			12.5	0.002^S^
Nulliparous	8 (8%)	25 (25%)		
Para 1-4	78 (78%)	69 (69%)		
Para ≥ 5	14 (14%)	6 (6%)		
Miscarriage			1.6	0.2^NS^
Yes	54 (54%)	45 (45%)		
No	46 (46%)	55 (55%)		
Gestational age			2.9	0.2^NS^
≤32 weeks	57 (57%)	66 (66%)		
33-36 weeks	39 (39%)	33 (33%)		
37-39 weeks	4 (4%)	1 (1%)		
Family history of DM			9.8	0.002^S^
Yes	67 (67%)	45 (45%)		
No	33 (33%)	55 (55%)		
Weight of previous baby			2.1	0.15^NS^
Normal	84 (94.4%)	74 (98.7%)		
Macrosomia	5 (5.6%)	1 (1.3%)		
Food type			6.0	0.04^S^
Animal source	1 (1%)	0 (0%)		
Plant source	0 (0%)	5 (5%)		
Both	99 (99%)	95 (95%)		

To evaluate the diagnostic performance of serum UA in identifying GDM, a ROC curve analysis was performed. The area under the curve (AUC) was 0.940, indicating excellent discriminative ability. The optimal cut-off value for UA was identified as 3.15 mg/dL, which yielded a sensitivity of 90% and a specificity of 80% for detecting GDM. This threshold was determined using Youden's index, which had a maximum value of 0.79, suggesting a high overall accuracy at this point (Figure 1).

RETRACTED

**Figure 1:** ROC curve for uric acid as a predictor for pregnancy outcome ROC: receiver operating characteristic

High random blood sugar levels of pregnant women were significantly related to GDM (p < 0.001). There was a highly significant association between high HbA1c levels of pregnant women and GDM (p < 0.001). A highly significant difference was observed between the mean serum UA level of the GDM group and the control group (p < 0.001). A significant association was found between elevated UA levels and GDM; 90 (90%) of pregnant women with GDM had serum UA levels of 3.15 mg/dL or more. Glycosuria was significantly related to GDM (p < 0.001); 19 (19%) of pregnant women with GDM had glycosuria (Table 4).

**Table 4:** Distribution of investigation findings according to study groups Calculated by the Chi-squared test S: significant; NS: not significant; GDM: gestational diabetes mellitus

Variable	Study groups		Χ^2^	p
	GDM	Control		
	No. (%)	No. (%)		
Random blood sugar level			48.4	<0.001^S^
Normal	61 (61.0%)	100 (100%)		
High	39 (39%)	0 (0%)		
HbA1c level			200.0	<0.001^S^
Normal	0 (0%)	100 (100%)		
High	100 (100%)	0 (0%)		
Serum uric acid level	4.4 ± 1.1	2.5 ± 0.6		<0.001^S^
<3.15 mg/dL	10 (10%)	89 (89%)		<0.001^S^
≥3.15 mg/dL	90 (90%)	11 (11%)		
Glycosuria			18.8	<0.001^S^
Yes	19 (19%)	0 (0%)		
No	81 (81%)	100 (100%)		

Increased age of pregnant women was significantly related to elevated serum UA levels (p = 0.001). Illiteracy was significantly higher among women with UA ≥ 3.15 (p < 0.05). No significant differences were observed between the study groups with regard to residence, blood groups, income, occupation, and house ownership (p > 0.05) (Table 5).

**Table 5:** Distribution of GDM women's sociodemographic characteristics according to serum uric acid level Calculated by the Chi-squared test S: significant; NS: not significant; GDM: gestational diabetes mellitus

Variable	Serum uric acid		Χ^2^	p
	<3.15 mg/dL	≥3.15 mg/dL		
	No. (%)	No. (%)		
Age, mean ± SD	28.1 ± 6.4	32.2 ± 5.8		<0.001^S^
18-35 years	85 (85.9%)	66 (65.3%)	11.4	0.001^S^
>35 years	14 (14.1%)	35 (34.7%)		
Residence			0.2	0.7^NS^
Rural	20 (20.2%)	23 (22.8%)		
Urban	79 (79.8%)	78 (77.2%)		
Blood groups			3.1	0.4^NS^
A	34 (34.3%)	46 (45.5%)		
B	24 (24.2%)	17 (16.8%)		
O	33 (33.3%)	30 (29.7%)		
AB	8 (8.1%)	8 (7.9%)		
Educational level			10.9	0.022^S^
Illiterate	32 (32.3%)	55 (54.5%)		
Read, write, & primary	51 (51.5%)	37(36.6%)		
Intermediate	8 (8.1%)	5 (5%)		
Secondary	4 (4%)	3 (3%)		
College and above	4 (4%)	1 (1%)		
Income			0.02	1.0^NS^
Not sufficient or marginally sufficient	15 (15.2%)	16 (15.8%)		
Sufficient	84 (84.8%)	85 (84.2%)		
Occupation			1.7	0.6^NS^
Housewife	86 (86.9%)	89 (88.1%)		
Student	5 (5.1%)	2 (2%)		
Governmental employee	4 (4%)	4 (4%)		
Non-governmental employee	4 (4%)	6 (5.9%)		
House ownership			0.7	0.7^NS^
Rented and others	23 (23.2%)	32 (31.7%)		
Partially owned	31 (31.3%)	35 (34.7%)		
Owned	45 (45.5%)	34 (33.7%)		

Increased BMI of pregnant women with GDM was significantly related to elevated serum UA level (p < 0.001). There was a significant association between increased gestational age of pregnant women and elevated serum UA level (p = 0.002). Multiparity was significantly associated with elevated UA level (p = 0.02). Family history of DM was significantly associated with elevated UA level (p = 0.003). No significant differences were observed between the study groups with regard to miscarriage and weight of previous baby (p > 0.05) (Table 6).

RETRACTED

**Table 6:** Distribution of GDM women's general characteristics according to serum uric acid level Calculated by the Chi-squared test *p-value is calculated by Fisher's exact test S: significant; NS: not significant; GDM: gestational diabetes mellitus; DM: diabetes mellitus

Variable	Serum uric acid		Χ^2^	p
	<3.15 mg/dL	≥3.15 mg/dL		
	No. (%)	No. (%)		
Body mass index			28.4	<0.001^S^*
Normal	29 (29.3%)	9 (8.9%)		
Overweight	49 (49.5%)	37 (36.6%)		
Obesity grade I	17 (17.2%)	39 (38.6%)		
Obesity grade II	4 (4%)	14 (13.9%)		
Obesity grade III	0 (0%)	2 (2%)		
Parity			7.4	0.02^S^
Nulliparous	23 (23.2%)	10 (9.9%)		
Para 1-4	69 (69.7%)	78 (77.2%)		
Para ≥ 5	7 (7.1%)	13 (12.9%)		
Miscarriage			1.3	0.3^NS^
Yes	45 (45.5%)	54 (53.5%)		
No	54 (54.5%)	47 (46.5%)		
Gestational age			11.5	0.002^S^*
≤32 weeks	71 (71.7%)	52 (51.5%)		
33-36 weeks	28 (28.3%)	44 (43.6%)		
37-39 weeks	0 (0%)	5 (5%)		
Family history of DM			8.8	0.003^S^
Yes	45 (45.5%)	67 (66.3%)		
No	54 (54.5%)	34 (33.7%)		
Weight of previous baby			1.1	0.4^NS^*
Normal	71 (94.7%)	87 (97.8%)		
Macrosomia	4 (5.3%)	2 (2.2%)		
Food type			6.2	0.03^S^*
Animal source	0 (0%)	1 (1%)		
Plant source	5 (5.1%)	0 (0%)		
Both	94 (94.9%)	100 (99%)		

The means of random blood sugar and HbA1c levels for pregnant women with GDM were significantly related to serum UA levels (p < 0.05) (Table 7).

**Table 7:** Distribution of investigation findings according to serum uric acid level Calculated by the t-test S: significant

Variable	Serum uric acid		t	p
	<3.15 mg/dL	≥3.15 mg/dL		
	Mean ± SD	Mean ± SD		
Random blood sugar level (mg/dL)	112.4 ± 27.0	163.4 ± 39.9	-10.5	<0.001^S^
HbA1c level (%)	5.1 ± 1.0	7.4 ± 1.2	-14.0	<0.001^S^

In this logistic regression model, higher serum UA levels were a strong and statistically significant predictor of the outcome, with each 1 mg/dL increase associated with a 30.7-fold increase in the odds (p < 0.001). Gestational age was also a significant predictor, where each additional week of gestation was linked to a 29.6% reduction in the odds (OR = 0.704, p = 0.005). BMI showed a borderline association (p = 0.063), suggesting that each unit increase in BMI may raise the odds by approximately 13.6%, although this did not reach statistical significance. Age had no meaningful effect on the outcome (p = 0.765). The model’s constant was not statistically significant (Table 8).

RETRACTED

**Table 8:** Multivariable logistic regression analysis of factors associated with gestational diabetes mellitus (Model 1) Calculated by binary logistic regression BMI: body mass index; CI: confidence interval; OR: odds ratio

Variable	OR	95% CI lower	95% CI upper	p-value
BMI	1.136	0.993	1.300	0.063
Gestational age	0.704	0.552	0.897	0.005
Age	0.987	0.906	1.075	0.765
Serum uric acid (mg/dL)	30.679	10.907	86.293	0.000

When UA was analyzed as a categorical variable rather than a continuous one, women with levels > 3.15 mg/dL had 122.8-fold higher odds of developing GDM compared to those with lower levels (p < 0.001), after adjusting for age, BMI, and gestational age. Each 1 kg/m² increase in BMI corresponded to a 28% rise in the odds of GDM (OR = 1.282, p = 0.001), while each additional week of gestation was associated with a 25% reduction in risk (OR = 0.750, p = 0.016). Age did not emerge as a significant predictor (p = 0.978) (Table 9).

**Table 9:** Multivariable logistic regression analysis of factors associated with gestational diabetes mellitus (Model 2) Calculated by binary logistic regression OR: odds ratio; CI: confidence interval; BMI: body mass index

Variable	OR	95% CI lower	95% CI upper	p-value
BMI	1.282	1.113	1.477	0.001
Gestational age	0.750	0.593	0.949	0.016
Age	1.001	0.920	1.090	0.978
Serum uric acid (mg/dL)	122.8	34.43	437.84	0.000

## Discussion

GDM is a common obstetrical disorder with a significant impact on maternal and fetal well-being. Assessing the role of serum UA level in pregnancy is important in the screening, diagnosis, and treatment of GDM [21].

The current study showed that increased age of pregnant women was significantly related to GDM. A recent systematic review and meta-analysis from China documented a linear relationship between increased age of pregnant women and GDM incidence [22]. The present study found a highly significant relationship between illiteracy among pregnant women and GDM. Illiteracy is associated with poor SES, which leads to decreased physical activity and health education, which all play a major role in the development of GDM [23].

RETRACTED

In this study, obesity, grand multiparity, and positive family history of GDM were significant risk factors for GDM. These findings are similar to the results of different recent studies in Saudi Arabia and Poland [24,25]. The current study showed a significant association between the lack of plant-based food intake and GDM. In the same direction, a review from Italy stated that a plant-based diet for pregnant women was helpful in the prevention of GDM [26].

The present study found a highly significant association between elevated serum UA levels and GDM. This finding coincides with the results of many recent studies conducted in Iraq and Iran, which revealed a significant relationship between elevated serum UA levels and pregnant women with GDM [27,28]. In this study, 90% of pregnant women with GDM had serum UA levels ≥ 3.15 mg/dL, a cut-off value determined from the ROC curve, which demonstrated 90% sensitivity and 80% specificity for identifying GDM. A recent prospective cohort study carried out in Egypt reported that 54.7% of pregnant women with GDM had elevated serum UA levels (>5 mg/dL) [29]. A 2025 observational study conducted at a hospital in India found that using a first-trimester serum UA cut-off > 3.4 mg/dL yielded a sensitivity of 74.7% and specificity of 82.6% for predicting GDM (area under the ROC (AU-ROC) = 0.832) [30]. Moreover, in the current study, after adjusting for age, BMI, and gestational age, higher serum UA remained a strong, statistically significant predictor of the outcome, with each 1 mg/dL increase associated with 30.7-fold higher odds (p < 0.001). Similarly, Patil and Bhattacharya [30] also reported that women with UA levels above 3.4 mg/dL had 14-fold higher odds of developing GDM (OR = 14.02; 95% CI: 4.28-45.92; p < 0.001). Differences in elevated serum UA prevalence between studies might be attributed to discrepancies in women's risk factors and the definition of elevation between various studies. However, some large-scale cohort studies such as those by Zhao et al. [17] and Li et al. [16] reported inconsistent findings, where serum UA measured in early pregnancy was not always a strong predictor of GDM after adjusting for confounders. These discrepancies may stem from differences in study design, timing of UA measurement, population characteristics, or diagnostic criteria. Khan et al. [15] documented that increased serum UA levels increased the risk of GDM and adverse pregnancy outcomes among pregnant women with GDM. In this study, high random blood sugar, HbA1c, and glycosuria levels of pregnant women were significantly related to GDM. These findings are in agreement with the results of different studies carried out in the Philippines and Ghana [1,31].

RETRACTED

Mechanistically, elevated UA may contribute to insulin resistance through several pathways. Experimental studies have shown that UA can directly inhibit insulin signaling in adipocytes and skeletal muscle cells by activating inflammatory pathways and oxidative stress [11]. Furthermore, UA reduces nitric oxide bioavailability, leading to endothelial dysfunction, which may impair insulin-mediated glucose uptake [12-14]. These biological effects may exacerbate the insulin resistance already present in pregnancy, tipping the balance toward hyperglycemia in susceptible individuals.

In this study involving 200 pregnant women, GDM was significantly associated with increased maternal age, illiteracy, higher BMI, grand multiparity, positive family history of diabetes, and lack of plant-based food intake. Elevated levels of random blood sugar, HbA1c, serum UA (≥3.15 mg/dL), and the presence of glycosuria were all significantly more frequent in women with GDM. Among women with GDM, those with elevated serum UA were more likely to be older, have higher BMI, and present at a later gestational age. Furthermore, a significant association was found between serum UA levels at a cut-off of 3.15 mg/dL and glycemic markers (random blood sugar and HbA1c) within the GDM group.

This study has several limitations. First, a small sample size and formal matching between cases and controls on age and BMI were not performed, although these variables, along with gestational age, were adjusted for in the multivariable logistic regression models. Second, dietary intake, physical activity, and renal function parameters such as serum creatinine were not measured or adjusted, which could have helped account for the influence of renal clearance on serum UA levels; however, women with known renal disease or on UA-altering medications were excluded. These unadjusted or partially adjusted confounders could potentially affect the robustness of our findings by influencing the observed strength of association between serum UA and GDM. Third, the study relied on self-reported sociodemographic and obstetric history, introducing a potential risk of recall bias. Fourth, although all GDM cases were diagnosed using the ADA 75 g OGTT criteria and all controls were confirmed free of GDM during the same pregnancy, in the absence of universal early pregnancy screening, a very small number of women-estimated at less than 5% of the control group-could theoretically have had undiagnosed GDM at another stage of gestation [32]. Fifth, the questionnaire used was designed by the research team and, while it underwent expert review and pilot testing, it was not a formally validated instrument. Sixth, the case-control design limits causal inference, and the facility-based recruitment may affect generalizability to the wider pregnant population. The laboratory procedures lacked detailed information on quality control or blinding, and the statistical analysis did not include multivariable models to assess the independent association between UA and GDM. Lastly, the 23.7% prevalence assumption used for sample size calculation was not based on local data, which may affect the robustness of the study's power estimation. Future studies should incorporate matched designs, direct renal function assessment, validated questionnaires, and longitudinal follow-up to better clarify temporal relationships and predictive value.

RETRACTED

## Conclusions

This study found that serum UA levels are significantly higher in pregnant women with GDM compared to healthy controls and are associated with glycemic markers (random blood sugar and HbA1c) within the GDM group. The optimal pregnancy-specific cut-off identified by ROC analysis was 3.15 mg/dL, providing 90% sensitivity and 80% specificity for predicting GDM, consistent with values reported in similar populations. These findings suggest that serum UA may serve both as a predictive marker for GDM development and as an indicator of metabolic disturbance after diagnosis.

Key limitations include the absence of direct renal function measurements, lack of dietary and physical activity data, and reliance on self-reported sociodemographic information, which may affect the robustness and generalizability of the results. Future research should confirm these findings in larger, matched cohorts with comprehensive adjustment for potential confounders.

## Appendices

**Table 10:** Questionnaire for the research assessment of serum uric acid levels among gestational diabetes patients in Erbil city Credits: Lezma Ghazy Qadir and Dr. Jwan Muhammad Zangana BMI: body mass index; DM: diabetes mellitus; RBS: random blood sugar

Code:	Phone number:
Name:	
Age in years:	
Residency:	1. Rural 2. Urban
Blood group:	1. A 2. B 3. O 4. AB
Educational level:	0. Illiterate 1. Read, write, & primary 2. Intermediate (7-9) years 3. Secondary (10-12) years 4. College and above
Income:	0. Not sufficient or marginally sufficient 1. Sufficient 2. Exceeds daily needs
Occupation	0. Housewife 1. Student 2. Governmental employee 3. Non-governmental employee
House ownership	0. Rented and others 1. Partially owned 2. Owned
Weight in kg (pre-pregnancy):	
Height in meters:	
BMI:	
Parity:	
Miscarriage:	
Family hx. of DM:	1. Yes 0. No
Gestational age in weeks:	
Weight of previous baby in kg:	
Type of food utilized:	Animal source Plant source Both
RBS (mg/dL) (postprandial)	
HbA1c	
Serum uric acid (mg/dL):	
Presence of glycosuria: if yes:	0. No 1. Yes: +1 +2 +3 +≥4
